This article has been retracted.

# Role of perceptual integration in pitch discrimination at high frequencies^a)^

**DOI:** 10.1121/10.0013429

**Published:** 2022-08-01

**Authors:** Anahita H. Mehta, Andrew J. Oxenham

**Affiliations:** Department of Psychology, University of Minnesota, Minneapolis, Minnesota 55455, USA

## Abstract

At very high frequencies, fundamental-frequency difference limens (F0DLs) for five-component harmonic complex tones can be better than predicted by optimal integration of information, assuming performance is limited by noise at the peripheral level, but are in line with predictions based on more central sources of noise. This study investigates whether there is a minimum number of harmonic components needed for such super-optimal integration effects and if harmonic range or inharmonicity affects this super-optimal integration. Results show super-optimal integration, even with two harmonic components and for most combinations of consecutive harmonic, but not inharmonic, components.

## 1. Introduction

Pitch and harmonicity are central properties of real-world sounds, including speech and music (Oxenham, 2018). Models of how pitch is extracted from both pure and complex tones have traditionally relied on either a timing code based on the phase-locking properties of the auditory nerve (Cariani and Delgutte, 1996; Meddis and O’Mard, 1997), a place code based on the tonotopic organization of the cochlea and auditory nerve (Cohen *et al*., 1995; Wightman, 1973), or a place-time code based on both phase locking and tonotopic organization (Cedolin and Delgutte, 2010; Shamma and Klein, 2000). For timing models, it is assumed that pitch coding is constrained by the upper frequency limit of phase locking. Although the extent of this upper limit is debated (Verschooten *et al*., 2019), it is generally believed that phase locking to the temporal fine structure (TFS) of stimuli is severely reduced or absent for frequencies above 8 kHz (Heinz *et al*., 2001; Recio-Spinoso *et al*., 2005). Accordingly, the degradation in pure-tone frequency discrimination at frequencies between 4 and 8 kHz has been attributed to a peripheral source, namely the degradation in auditory-nerve phase locking (e.g., Moore and Ernst, 2012).

When multiple pure tones form consecutive components of a harmonic series, listeners typically perceive a pitch corresponding to the fundamental frequency (F0) of the complex, even when no energy is present at the F0 itself. Lau *et al*. (2017) reported good F0 discrimination for complex tones with an F0 of 1400 Hz, even though the complexes contained only harmonics above 8 kHz. The results were not due to peripheral interactions between the individual harmonics, causing beats or envelope fluctuations at the F0, as the F0 difference limens (F0DLs) remained the same when alternating components were presented to opposite ears (Lau *et al*., 2017).

Lau *et al*. (2017) compared the obtained F0DLs with predictions based on the frequency difference limens (FDLs) from the individual components presented in isolation. Using signal detection theory (Green and Swets, 1966), F0DL predictions were calculated based either on the assumption that performance is limited by neural coding noise that is applied before the information from each component is combined (early- or peripheral-noise model) or on the assumption that performance is limited by a neural coding noise that is applied after the information from each component is combined (late- or central-noise model). Lau *et al*. (2017) found that F0DLs were significantly lower (better) than the optimal-integration predictions of the early-noise model and that performance was instead well predicted by the central-noise model. The results suggested a central, rather than peripheral, limiting factor to high-frequency pitch discrimination, which in turn suggests that peripheral phase locking may not be responsible for limiting performance.

Attempts to replicate parts of the Lau *et al*. (2017) study have been met with mixed success (Gockel *et al*., 2020; Gockel and Carlyon, 2018). Gockel and Carlyon (2018) also found similar F0DLs for high-frequency complex tones presented diotically and dichotically (all components to both ears or alternating components to opposite ears, respectively), confirming the lack of influence of temporal-envelope cues, but their F0DLs were lower (better) than in the original study by about a factor of 2. Gockel *et al*. (2020) replicated the basic finding of better F0DLs than FDLs at high frequencies, but their high-frequency FDLs for components at 8.4 and 9.8 kHz (harmonics 6 and 7 of 1.4 kHz) were already so low [~2%, a factor of 3–7 lower than those reported by Lau *et al*. (2017)] that the difference between the FDLs and F0DLs was no longer significantly different from that predicted by optimal integration assuming peripheral noise.

The current study addresses these apparent discrepancies in two ways. First, we attempted to replicate the original findings of Lau *et al*. (2017) to test their reliability. We compared FDLs and F0DLs at high frequencies for tones that were either in harmonic relationship or were all shifted by 0.5F0 Hz to produce inharmonic complex tones that maintained the same component spacing as the harmonic complex tones. The hypothesis was that perceptual integration that was better than expected based on peripheral limitations, if found at all, should be limited to the harmonic tones, as these would be most likely to elicit a central representation of F0 (e.g., Allen *et al*., 2022; Bendor and Wang, 2005). Second, we provided stronger tests of perceptual integration by testing various combinations of two, three, and four components, rather than just the five components (harmonics 6–10) tested in the previous studies. The rationale for this extension was to determine whether any super-optimal integration for harmonic tones, and any difference between the integration of harmonic and inharmonic tones, generalized to conditions beyond the original five-component complexes tested in all the previous studies. Pitch salience is known to increase with increasing number of harmonic components up to about 4 or 5 (e.g., Laguitton *et al*., 1998); therefore, it is possible that super-optimal integration only occurs when a minimum number of components are present.

## 2. Methods

### 2.1 Participants

Thirty-six participants were initially recruited, none of whom had previously taken part in the earlier study (Lau *et al*., 2017). Sixteen normal-hearing participants (11 female, 5 male) between 19 and 27 years of age (mean: 22 years) with audiometric thresholds no greater than 15 dB hearing level (HL) at octave frequencies from 250 to 8000 Hz participated in the actual study after passing all screening tasks. The musical experience of these 16 participants ranged from 0 to 20 years (mean: 6 years). No participant reported a history of neurological or hearing disorders. Written informed consent was provided by each participant, and all participants were compensated for their time. The experiment was conducted at the University of Minnesota–Twin Cities. The protocol was approved by the Institutional Review Board of the University of Minnesota.

### 2.2 Screening

As the experiments involved tones up to 16 kHz, all participants were required to pass a high-frequency hearing screening extending to 16 kHz and a high-frequency pitch-discrimination screening to take part in the main experiment. For the first screening, detection thresholds were measured for pure tones at 14 and 16 kHz in the same background noise as was used in the main experiments. The background noise was threshold-equalizing noise (TEN) (Moore *et al*., 2000) extending from 20 to 22 000 Hz, at a level of 45 dB sound pressure level (SPL) per estimated equivalent rectangular bandwidth (ERB) of the auditory filter as defined at 1 kHz (Glasberg and Moore, 1990). Thresholds were measured using an adaptive three-interval three-alternative forced-choice procedure with a three-down one-up rule that tracks the 79.4% point on the psychometric function (Levitt, 1971). The average of three such runs defined the threshold for each participant. Twelve of the initial 36 participants failed the hearing screening.

For the second screening, F0DLs and FDLs were measured for the same harmonic-tone stimuli as used in experiment 1 of this study, but without level randomization and without background noise. Thresholds were measured using a two-interval two-alternative forced-choice procedure similar to that used in the main experiment. Listeners performed two runs for each stimulus condition and were required to have average F0DLs of less than 20%. Eight additional participants were excluded due to failing this stage of the screening. The musical experience of these eight participants ranged from 0 to 14 years (median: 6 years).

### 2.3 Sound presentation and calibration

All test sessions took place in a double-walled sound-attenuating booth. The stimuli were presented binaurally (diotically) via Sennheiser (Wedemark, Germany) HD 650 headphones, which have an approximately diffuse-field response, so the sound pressure levels specified are approximate equivalent diffuse-field levels. The experimental stimuli were generated digitally and presented via a LynxStudio (Costa Mesa, CA) e22 soundcard with 24-bit resolution at a sampling rate of 48 kHz.

### 2.4 Experiments

All 16 subjects who passed both screenings completed all experiments described below. Due to the screening procedure, they had all undertaken at least 1 h of training with high-frequency F0 and frequency discrimination. The order of experiments (experiments 1 and 2; harmonic and inharmonic) was randomized across participants. The entire study took about 4–5 sessions of 2 h each per participant.

#### 2.4.1 Experiment 1

This experiment involved direct replications of experiment 1 (harmonic tones) and experiment 5 (inharmonic tones) of Lau *et al*. (2017), but tested in the same participants and in counterbalanced order. For the harmonic conditions, we measured FDLs for pure tones corresponding to the sixth to tenth harmonics of 1400 Hz and the F0DLs for the complex tone consisting of the same harmonics in random phase. For the inharmonic conditions, FDLs and F0DLs were measured for tones corresponding to multiples of 6.5, 7.5, 8.5, 9.5, and 10.5 of the F0 (1400 Hz). For the complex tones only, the inner components (harmonics 7–9 or 7.5–9.5) were presented at 55 dB SPL, and the outer components (6 and 10 or 6.5 and 10.5) were presented at 49 dB SPL per component to reduce spectral edge cues (Kohlrausch and Houtsma, 1992), as shown in Fig. 1. The pure tones were always presented at 55 dB SPL. Additionally, the level of each tone component was independently roved by ±3 dB to reduce possible level cues. Finally, all the stimuli were embedded in TEN, presented at 45 dB SPL within the ERB around 1 kHz to reduce the audibility of potential distortion products. The threshold in each condition for each participant was defined as the geometric mean of the thresholds obtained across four runs. The thresholds were estimated using a two-interval two-alternative forced-choice paradigm with a three-down one-up adaptive procedure. Each trial consisted of a 210-ms tone followed by a 500-ms gap and a second 210-ms tone. The background noise was gated on 200 ms before the first tone and gated off 100 ms after the end of the second tone. The participants had to indicate which interval had the higher pitch for all tasks in this study. Feedback was provided after each trial. The starting value of the change in pure-tone frequency or complex-tone F0 (Δf or ΔF0, respectively) was 20%, with the frequencies of the two tones geometrically centered on the nominal test frequency or F0. Initially, the value of Δf or ΔF0 increased or decreased by a factor of 2. The step size was decreased to a factor of 1.41 after the first two reversals and to a factor of 1.2 after the next two reversals. An additional six reversals occurred at the smallest step size, and the difference limen (DL) was calculated as the geometric mean of the Δf or ΔF0 values at those last six reversal points. The presentation order of the conditions was randomized for each participant.

#### 2.4.2 Experiment 2

This experiment was designed to test perceptual integration for multiple combinations of harmonic and inharmonic tones with the same F0 (1400 Hz) and components (harmonics 6–10) as were used in experiment 1. For the harmonic conditions, the combinations tested were harmonics 6 and 7, 6–8, 6–9, 9 and 10, 8–10, and 7–10. The inharmonic conditions were the same as the harmonic conditions in experiment 2 but incremented by 0.5 F0. All components were presented at 55 dB SPL. All other details of the stimuli and procedure were the same as in experiment 1.

### 2.5 Analyses

Predictions of the F0DLs from the FDLs of the individual components were calculated using an approach based on signal detection theory (Green and Swets, 1966), as was done by Lau *et al*. (2017). The F0DL estimate based on peripheral noise assumed that performance is limited by noise due to peripheral coding variability, such as the limitations of phase locking, before the integration of information (“early-noise model”). The F0DL estimate based on central noise assumed that information from individual components is integrated without limitations of peripheral noise and is instead limited by a central noise imposed after the information from the individual components has been integrated (“late-noise model”).

## 3. Results

### 3.1 Experiment 1: Observed and predicted F0DLs for harmonic and inharmonic tones

The geometric mean FDLs and F0DLs from experiment 1 are shown in Fig. 2 as open circles, with harmonic tones in orange and inharmonic tones in purple. Predicted F0DLs from the early-noise and late-noise models are shown as filled squares and diamonds, respectively.

Considering first the pure-tone data, a repeated-measures analysis of variance (ANOVA) on the log-transformed FDLs with harmonicity and harmonic number (rounding down the inharmonic numbers) as within-subjects factors confirmed no significant main effect of, and no interaction with, harmonicity (*F*_1,15_ = 0.117, *p* = 0.74, and *F*_4,60_ = 1.03, *p* = 0.39, respectively) but showed a main effect of harmonic number (*F*_4,60_ = 12.03, *p* < 0.001), reflecting the increase in FDL with increasing harmonic number between 6 and 8. The same statistical conclusions were reached when the inharmonic numbers were rounded up instead of down (e.g., harmonic 6.5 was grouped with harmonic 7).

In contrast to the lack of effect with the pure tones, there was a significant difference between F0DLs for the harmonic and inharmonic complex tones (paired *t*-test on the log-transformed F0DLs, *t*_15_ = −3.16, *p* = 0.012), reflecting the fact that the mean F0DL in the inharmonic condition was nearly twice that in the harmonic condition. Because the early- and late-noise model predictions are derived from the same data, they are not independent. For that reason, they were compared with the observed data in separate analyses.

Considering first the predictions from the early-noise (peripheral) model, a repeated-measures ANOVA on the F0DLs with factors of harmonicity (harmonic vs inharmonic) and measure type (predicted vs observed) found no main effect of harmonicity (*F*_1,15_ = 1.51, *p* = 0.24) but a main effect of measure type (*F*_1,15_ = 6.35, *p* = 0.02) and a significant interaction (*F*_1,15_ = 5.92, *p* = 0.03). *Post hoc* pairwise comparisons showed a significant difference between observed and predicted thresholds for harmonic complex tones (*p* = 0.006) but no significant difference between observed and predicted thresholds for inharmonic complex tones (*p* = 0.544). Thus, the peripheral (early-noise) model was able to predict F0DLs for the inharmonic but not the harmonic complex tones.

Considering next the predictions from the late-noise (central) model, a repeated-measures ANOVA on the F0DLs with factors of harmonicity (harmonic vs inharmonic) and measure type (predicted vs observed) again found no main effect of harmonicity (*F*_1,15_ = 1.66, *p* = 0.22), but a main effect of measure type (*F*_1,15_ = 21.4, *p* < 0.001), and a significant interaction (*F*_1,15_ = 6.55, *p* = 0.02). *Post hoc* pairwise comparisons showed no significant difference between observed and predicted thresholds for harmonic complex tones (*p* = 0.75) and a significant difference between observed and predicted thresholds for inharmonic complex tones (*p* < 0.001). Thus, the central (late-noise) model was able to predict F0DLs for harmonic but not the inharmonic complex tones—the opposite of the pattern observed for the peripheral (early-noise) model.

In the harmonic-tone conditions, there was greater improvement from individual FDLs to complex-tone F0DLs than can be predicted even with optimal integration of information, if it is assumed that information is limited peripherally. The data were, however, consistent with predictions from a model assuming optimal integration of information with a central noise limiting performance. The opposite was true for the inharmonic-tone conditions, with peripheral-noise predictions providing a better match to the data. This difference in perceptual integration between harmonic and inharmonic tones was due to significantly poorer F0DLs for inharmonic than for harmonic complex tones.

### 3.2 Experiment 2: Observed and predicted F0DLs as a function of number of components

The question addressed here was whether the same patterns of perceptual integration can be generalized beyond the five-component conditions tested in experiment 1 and by Lau *et al*. (2017). Figure 3 shows mean observed F0DLs for various combinations of two, three, and four consecutive harmonic and inharmonic (shifted) components, along with the predictions for each combination, based on the pure-tone FDLs in experiment 1 from the same participants. As in experiment 1, two separate repeated-measures ANOVAs were conducted on the F0DLs, one for the peripheral predictions, based on the early-noise model, and the other for the central predictions, based on the late-noise model. The factors were harmonicity (harmonic or inharmonic), measure type (observed or predicted), and component combination (6–7, 6–8, 6–9, 9–10, 8–10, or 7–10).

For the peripheral (early-noise) model, we found no main effect of harmonicity (*F*_1,15_ = 2.12, *p* = 0.16), a main effect of measure type (*F*_1,15_ = 14.3, *p* = 0.002), and a main effect of component combination (*F*_5,75_ = 18.6, *p* < 0.001). We also found significant interactions between harmonicity and measure type (*F*_1,15_ = 9.72, *p* = 0.008) and between harmonicity and component combination (*F*_5,75_ = 6.56, *p* < 0.001) but no other significant interactions. *Post hoc* pairwise comparisons showed no significant difference between observed and peripheral-predicted F0DLs for inharmonic complex tones (*p* = 0.08) but a significant difference between observed and peripheral-predicted F0DLs for harmonic complex tones (*p* < 0.001).

For the central (late-noise) model, we found no main effect of harmonicity (*F*_1,15_ = 2.43, *p* = 0.14), a main effect of measure type (*F*_1,15_ = 7.72, *p* = 0.015), and a main effect of component combination (*F*_5,75_ = 23.6, *p* < 0.001). We also found a significant interaction between harmonicity and measure type (*F*_1,15_ = 12.04, *p* = 0.004) and a significant interaction between harmonicity and component combination (*F*_5,75_ = 7.06, *p* < 0.001). No other interactions reached significance. *Post hoc* pairwise comparisons showed no significant difference between observed and central-predicted F0DLs for the harmonic complex tones (*p* = 0.49) but significant differences between observed and central-predicted F0DLs for the inharmonic complex tones (*p* < 0.001).

An additional analysis was conducted to investigate the effect of the number of components and the lowest component included. Two separate repeated-measures ANOVAs were conducted on the observed harmonic and inharmonic F0DLs. The factors were number of components (two, three, or four) and the fixed component (either six or ten). For the harmonic F0DLs, we found a main effect of fixed component (*F*_1,15_ = 17.2, *p* < 0.001), a main effect of number of components (*F*_2,30_ = 28.45, *p* < 0.001), and no significant interaction (*F*_2,30_ = 1.98, *p* = 0.156). For the inharmonic F0DLs, we also found a main effect of fixed component (*F*_1,15_ = 5.455, *p* = 0.034), a main effect of number of components (*F*_2,30_ = 25.61, *p* < 0.001), and no significant interaction (*F*_2,30_ = 1.51, *p* = 0.238).

The results showed that perceptual integration occurs with as few as two adjacent components and that the pattern observed in experiment 1 with five components holds for combinations of two, three, and four components, with integration consistent with central limitations (late-noise model) occurring for harmonic complex tones and integration consistent with peripheral limitations (early-noise model) occurring for inharmonic (shifted) complex tones.

## 4. Discussion

In experiment 1, we replicated the findings of Lau *et al*. (2017), with F0DLs for high-frequency complex tones considerably lower than the FDLs for the individual constituent components, and also showed that F0DLs were significantly lower (better) for harmonic than for inharmonic (shifted) complex tones in the same participants. Critically, we confirmed that obtained F0DLs for the harmonic complex tones were significantly different (better) than predicted by optimal integration of information, assuming an early-noise model, but were not significantly different from predictions based on optimal integration of information assuming a late-noise model. The opposite pattern was found for inharmonic tones. Experiment 2 showed that this pattern of perceptual integration (and difference between harmonic and inharmonic tones) extends to conditions with various combinations of two, three, and four consecutive harmonics.

The finding of substantially poorer F0DLs for inharmonic (shifted) complexes than for harmonic complexes at high frequencies is different from what is observed at lower frequencies, where the differences between harmonic and shifted inharmonic F0DLs are generally quite small (McPherson and McDermott, 2018; Micheyl *et al*., 2010). The effect of absolute frequency may occur because at low frequencies, both FDLs and F0DLs are very similar (often <1%) and are likely limited by the resolution of individual components; in contrast, at the very high frequencies tested here, individual FDLs are much poorer than F0DLs, meaning that performance for complex tones likely relies more strongly on higher-level percepts, such as pitch, and so may be more affected by inharmonicity, which weakens the percept of pitch. A difference between detection thresholds (Hafter and Saberi, 2001; McPherson *et al*., 2022) as well as discrimination thresholds (Carlyon and Stubbs, 1989) using harmonic and inharmonic complex tones at lower F0s has been reported in the presence of background noise. However, as our complex tones were all presented well above detection threshold, the differences in discrimination thresholds between harmonic and inharmonic tones seem unlikely to be solely due to improved detectability of the harmonic tones. Finally, although the inharmonic-complex F0DLs were not significantly different from the peripheral-noise model predictions, there was a trend for them to lie between the predictions of the two models. This trend may be due to the residual, albeit weak and potentially ambiguous, pitch elicited by inharmonic complex tones (de Boer, 1956; Patterson and Wightman, 1976).

Gockel *et al*. (2020) used a similar paradigm to that of experiment 1 in both this study and that of Lau *et al*. (2017). The main stimulus difference was the use of continuous diotic TEN background noise instead of the gated TEN used here and by Lau *et al*. (2017). Although it is unlikely that this difference would contribute to the difference in thresholds, there is a possibility that the continuous noise might have been less distracting than gated noise due to the lack of noise onsets and offsets. Another potentially important difference was that their participants appear to have been much more practiced at listening to very high-frequency tones. The more extensive practice of the participants of Gockel *et al*. may explain why their pure-tone FDLs for tones above 8 kHz were a factor of 3–7 times lower (better) than those reported by Lau *et al*. (2017) and those reported here. To determine whether some of the individual differences and differences between studies in the FDLs could be due to differences in musical training, a correlation was conducted between FDLs for the lowest harmonic (sixth) in experiment 1 and years of musical training. No significant correlation was obtained (Pearson’s *r*_15_ = 0.068, *p* = 0.803), consistent with the findings of Lau *et al*. (2017), who also found no correlation between FDLs and years of musical experience.

The harmonic-tone F0DLs reported by Gockel *et al*. (2020) were only a factor 3 or so lower than those found by Lau *et al*. (2017) and here in experiment 1, meaning that the ratio between the FDLs and F0DLs of Gockel *et al*. (2020) was not as great as found by either Lau *et al*. (2017) or here and was not significantly greater than predicted by optimal integration under the early-noise model. The fact that extensive practice may lead to considerably lower high-frequency FDLs could in itself be taken as support for the idea that central, rather than peripheral, noise limits high-frequency pitch discrimination, as it seems more likely that any neural plasticity induced by practice will affect central, rather than auditory-nerve, representations of the sounds.

In summary, the results presented here confirm that perceptual integration of information from high-frequency harmonics can exceed that predicted by optimal integration of information when the information is limited by a peripheral noise source (such as auditory-nerve phase locking) and is instead consistent with a more central limiting noise source. The results also show that this integration occurs when as few as two consecutive harmonics are present, and even when the harmonics are all above 10 kHz (seen in the results of harmonics 10–8), and thus unlikely to provide any phase-locked information (Verschooten *et al*., 2018; Verschooten *et al*., 2019). The fact that only harmonic, and not inharmonic, tones exhibit this “super-optimal integration” also argues for the importance of central representations, possibly involving cortical neurons sensitive to harmonicity (Feng and Wang, 2017) and/or pitch (Allen *et al*., 2022; Bendor and Wang, 2005).

## Figures and Tables

**Fig. 1.** Schematic of complex-tone stimuli used in experiment 1. The *x* axis shows the frequency of the components for the harmonic (left) and shifted-harmonic (right) conditions. The edge components were lower in amplitude by 6 dB to reduce potential spectral edge pitch cues.

**Fig. 2.** Mean F0DLs (left of the vertical dashed line) and FDLs (right of dashed line) for experiment 1 (*n* = 16). Error bars represent ±1 standard error of the mean (SEM). The filled squares represent peripheral predicted F0DLs, based on the early-noise model. The filled diamonds represent central predicted F0DLs, based on the late-noise model. The observed thresholds are shown by the open circles. The orange symbols represent harmonic conditions (integer multiples of 1400 Hz), and the purple symbols represent inharmonic conditions (shifted upward by 0.5F0).

**Fig. 3.** Mean F0DLs for various combinations of two, three, and four consecutive components in experiment 2 (*n* = 16). Error bars represent ±1 SEM. Harmonic and inharmonic (shifted) conditions are shown in the left and right panel, respectively. The *x* axis shows the harmonics present in each condition. The filled squares represent peripheral predicted F0DLs, based on the early-noise model. The filled diamonds represent central predicted F0DLs, based on the late-noise model. The observed thresholds are shown by the open circles.

## References

[R1] AllenEJ, MesikJ, KayKN, and OxenhamAJ (2022). “Distinct representations of tonotopy and pitch in human auditory cortex,” J. Neurosci 42, 416–434.3479941510.1523/JNEUROSCI.0960-21.2021PMC8802918

[R2] BendorD, and WangX (2005). “The neuronal representation of pitch in primate auditory cortex,” Nature 436, 1161–1165.1612118210.1038/nature03867PMC1780171

[R3] CarianiPA, and DelgutteB (1996). “Neural correlates of the pitch of complex tones. I. Pitch and pitch salience,” J. Neurophysiol 76, 1698–1716.889028610.1152/jn.1996.76.3.1698

[R4] CarlyonRP, and StubbsRJ (1989). “Detecting single-cycle frequency modulation imposed on sinusoidal, harmonic, and inharmonic carriers,” J. Acoust. Soc. Am 85, 2563–2574.

[R5] CedolinL, and DelgutteB (2010). “Spatiotemporal representation of the pitch of harmonic complex tones in the auditory nerve,” J. Neurosci 30, 12712–12724.2086137610.1523/JNEUROSCI.6365-09.2010PMC2957107

[R6] CohenMA, GrossbergS, and WyseLL (1995). “A spectral network model of pitch perception,” J. Acoust. Soc. Am 98, 862–879.764282510.1121/1.413512

[R7] de BoerE (1956). “Pitch of inharmonic signals,” Nature 178, 535–536.1335879010.1038/178535a0

[R8] FengL, and WangX (2017). “Harmonic template neurons in primate auditory cortex underlying complex sound processing,” Proc. Natl. Acad. Sci. U.S.A 114, E840–E848.2809634110.1073/pnas.1607519114PMC5293092

[R9] GlasbergBR, and MooreBCJ (1990). “Derivation of auditory filter shapes from notched-noise data,” Hear. Res 47, 103–138.222878910.1016/0378-5955(90)90170-t

[R10] GockelHE, and CarlyonRP (2018). “Detection of mistuning in harmonic complex tones at high frequencies,” Acta Acust. united Acust 104, 766–769.

[R11] GockelHE, MooreBCJ, and CarlyonRP (2020). “Pitch perception at very high frequencies: On psychometric functions and integration of frequency information,” J. Acoust. Soc. Am 148, 3322–3333.3326139210.1121/10.0002668PMC7613188

[R12] GreenDM, and SwetsJA (1966). Signal Detection Theory and Psychophysics, Signal Detection Theory and Psychophysics (Wiley, Oxford, UK), pp. xi, 455.

[R13] HafterER, and SaberiK (2001). “A level of stimulus representation model for auditory detection and attention,” J. Acoust. Soc. Am 110, 1489–1497.1157235910.1121/1.1394220

[R14] HeinzMG, ColburnHS, and CarneyLH (2001). “Evaluating auditory performance limits: I. One-parameter discrimination using a computational model for the auditory nerve,” Neural Comput. 13, 2273–2316.1157099910.1162/089976601750541804

[R15] KohlrauschA, and HoutsmaAJM (1992). “Pitch related to spectral edges of broadband signals [and discussion],” Philos. Trans. R. Soc. London, Ser. B: Biol. Sci 336, 375–382.135437710.1098/rstb.1992.0071

[R16] LaguittonV, DemanyL, SemalC, and Liégeois-ChauvelC (1998). “Pitch perception: A difference between right- and left-handed listeners,” Neuropsychologia 36, 201–207.962218510.1016/s0028-3932(97)00122-x

[R17] LauBK, MehtaAH, and OxenhamAJ (2017). “Superoptimal perceptual integration suggests a place-based representation of pitch at high frequencies,” J. Neurosci 37, 9013–9021.2882164210.1523/JNEUROSCI.1507-17.2017PMC5597982

[R18] LevittH (1971). “Transformed up-down methods in psychoacoustics,” J. Acoust. Soc. Am 49, 467–477.5541744

[R19] McPhersonMJ, GraceRC, and McDermottJH (2022). “Harmonicity aids hearing in noise,” Atten. Percept. Biophys 84, 1016–1042.10.3758/s13414-021-02376-0PMC880341135102502

[R20] McPhersonMJ, and McDermottJH (2018). “Diversity in pitch perception revealed by task dependence,” Nat. Hum. Behav 2, 52–66.3022120210.1038/s41562-017-0261-8PMC6136452

[R21] MeddisR, and O’MardL (1997). “A unitary model of pitch perception,” J. Acoust. Soc. Am 102, 1811–1820.930105810.1121/1.420088

[R22] MicheylC, DivisK, WrobleskiDM, and OxenhamAJ (2010). “Does fundamental-frequency discrimination measure virtual pitch discrimination?,” J. Acoust. Soc. Am 128, 1930–1942.2096836510.1121/1.3478786PMC2981110

[R23] MooreBCJ, and ErnstSMA (2012). “Frequency difference limens at high frequencies: Evidence for a transition from a temporal to a place code,” J. Acoust. Soc. Am 132, 1542–1547.2297888310.1121/1.4739444

[R24] MooreBCJ, HussM, VickersDA, GlasbergBR, and AlcántaraJI (2000). “A test for the diagnosis of dead regions in the cochlea,” Br. J. Audiol 34, 205–224.1099745010.3109/03005364000000131

[R25] OxenhamAJ (2018). “How we hear: The perception and neural coding of sound,” Annu. Rev. Psychol 69, 27–50.2903569110.1146/annurev-psych-122216-011635PMC5819010

[R26] PattersonRD, and WightmanFL (1976). “Resiude pitch as a function of component spacing,” J. Acoust. Soc. Am 59, 1450–1459.93987810.1121/1.381034

[R27] Recio-SpinosoA, TemchinAN, van DijkP, FanY-H, and RuggeroMA (2005). “Wiener-kernel analysis of responses to noise of chinchilla auditory-nerve fibers,” J. Neurophysiol 93(6), 3615–3634.1565953210.1152/jn.00882.2004

[R28] ShammaS, and KleinD (2000). “The case of the missing pitch templates: How harmonic templates emerge in the early auditory system,” J. Acoust. Soc. Am 107, 2631–2644.1083038510.1121/1.428649

[R29] VerschootenE, DesloovereC, and JorisPX (2018). “High-resolution frequency tuning but not temporal coding in the human cochlea,” PLoS Biol. 16, e2005164.3032116610.1371/journal.pbio.2005164PMC6201958

[R30] VerschootenE, ShammaS, OxenhamAJ, MooreBCJ, JorisPX, HeinzMG, and PlackCJ (2019). “The upper frequency limit for the use of phase locking to code temporal fine structure in humans: A compilation of viewpoints,” Hear. Res 377, 109–121.3092768610.1016/j.heares.2019.03.011PMC6524635

[R31] WightmanFL (1973). “The pattern-transformation model of pitch,” J. Acoust. Soc. Am 54, 407–416.475901410.1121/1.1913592

